# Development and Characterization of Biodegradable Composite Films Based on Gelatin Derived from Beef, Pork and Fish Sources

**DOI:** 10.3390/foods2010001

**Published:** 2012-12-31

**Authors:** Zainal A. Nur Hanani, Eddie Beatty, Yrjo H. Roos, Mick A. Morris, Joseph P. Kerry

**Affiliations:** 1 Department of Food Technology, Faculty of Food Science and Technology, University Putra Malaysia, 43400 UPM Serdang, Selangor, Malaysia; E-Mail: hanani@food.upm.edu.my; 2 Food Packaging Group, School of Food and Nutritional Sciences, University College Cork, National University of Ireland, Cork, Ireland; E-Mail: e.beatty@ucc.ie; 3 School of Food and Nutritional Sciences, University College Cork, National University of Ireland, Cork, Ireland; E-Mail: Yrjo.Roos@ucc.ie; 4 Department of Chemistry, University College Cork, National University of Ireland, Cork, Ireland; E-Mail: M.A.Morris@ucc.ie

**Keywords:** gelatin, composite films, biodegradable, mechanical properties, barrier properties, FTIR

## Abstract

The objectives of this study were to develop composite films using various gelatin sources with corn oil (CO) incorporation (55.18%) and to investigate the mechanical and physical properties of these films as potential packaging films. There were increases (*p* < 0.05) in the tensile strength (TS) and puncture strength (PS) of films when the concentration of gelatin increased. The mechanical properties of these films were also improved when compared with films produced without CO. Conversely, the water barrier properties of composite films decreased (*p* < 0.05) when the concentration of gelatin in composite films increased. Comparing with pure gelatin films, water and oxygen barrier properties of gelatin films decreased when manufactured with the inclusion of CO.

## 1. Introduction

Biopolymers, based on carbohydrates and proteins, have been extensively studied to develop edible/biodegradable films with more versatile properties [1]. However, biopolymer films are limited in terms of usage, as they possess strong hydrophilic characteristics which make them poor water vapour barriers. Many studies have been conducted as a means of attempting to improve the mechanical and barrier properties of biopolymer films by incorporation of secondary polymer components to produce composite films [2,3,4,5,6,7,8,9]. Composite films manufactured by blending two or more polymers can be expected to have improved or modified mechanical and barrier properties [9]. The mechanical and barrier properties of composite films are strongly dependent upon the component polymer characteristics and their compatibility [2,9].

Generally, protein-based films offer better mechanical and barrier properties than those manufactured from polysaccharides [10]. This is primarily because of the specific structure that proteins possess and their ability to form strong intermolecular covalent, ionic and hydrogen bonds, thereby allowing them to form numerous peptide and amide linkages [11,12,13,14]. Generally, films manufactured using lipids have been shown to be good water vapour barriers; but have also been shown to have negative visual properties and be prone to brittleness, thereby reducing their potential commercial applications [6,15,16]. Lipids; comprised of waxes, fats and oils, have been mixed with protein or polysaccharides-based films to improve flexibility, coating characteristics, or to prevent sticking during the cooking of food products [17,18]. From all the commercial oils assessed, corn oil has been shown to be one of the most effective in decreasing the water vapour permeability of polysaccharide- and protein-based films [6,19,20]. 

In addition to lipid incorporation, altering the pH of film-forming solutions may also be one of the many approaches required to improve functional properties of biopolymer films [6,21,22,23,24]. According to Wang *et al.* [6], higher pH gelatin solutions were shown to produce optimal film properties such as improved water barrier and mechanical properties. These authors proposed that the optimal film-forming condition for gelatin films using response surface methodology was a pH of 10.54 and an oil level of 55.18% (w/w). While these conditions were determined through experimental modelling, no experimental studies were carried out to assess these conditions on edible/biodegradable film formation using gelatin. 

In our previous study [25], films manufactured from gelatin derived from beef, pork and fish sources with different concentration (4%–8%) have been developed and demonstrated some commercial usage. Therefore, the objectives of this study were to develop gelatin composite films derived from various sources using a pH of 10.54 and an oil concentration of 55.18% (as outlined by Wang *et al.* [6]), and compare the properties of these films with the gelatin films obtained by Nur Hanani *et al.* [25].

## 2. Experimental Section

### 2.1. Materials

Beef skin gelatin (Bloom 220), pork skin gelatin (Bloom 225) and fish skin gelatin from warm water Tilapia (Bloom 240) were purchased from Healan Ingredients Ltd. (York, England). Corn oil and glycerol were obtained from Sigma Aldrich Co. (St. Louis, MO, USA). For pH adjustment, NaOH was obtained in pellet form and lactic acid was obtained from Merck (Darmstadt, Germany) and May & Baker Ltd. (Dagenham, England), respectively.

### 2.2. Film Preparation

Gelatin powders were solubilised in distilled water at concentrations between 4%–8% (w/v). Glycerol was added as a plasticizer at a constant glycerol/gelatin powder ratio of 2:5 (w/w). Corn oil (CO) was introduced into all gelatin solutions at a set concentration of 55.18% (w/w), in accordance with those recommendations proposed by Wang *et al.* [6]. Dispersions were adjusted to a pH of 10.54 using 1 M NaOH or lactic acid, again following guidelines described by Wang *et al.* [6]. All solutions were stirred using a magnetic stirrer hotplate and heated to 80 °C for 30 min. Dispersions were homogenized in three passes at 480 bar (first stage at 450 bar, second stage at 30 bar) using an APV homogenizer 2000 series (APV, Alberslund, Denmark). Subsequently, films were cast by pouring solutions onto levelled circular Teflon-coated Perspex plates and dried for 24 h at 50% ± 5% relative humidity (RH) and at a temperature of 23 ± 2 °C. The films were peeled from the plates and cut prior to testing. 

### 2.3. Film Morphology

Scanning electron microscopy (SEM) was used to investigate the morphology of the films using JSM-5510 (SEM, JEOL Ltd., Tokyo, Japan) at 5.0 kV. Film samples were cut into appropriate-sized samples and mounted on stubs using double-sided adhesive tape. Prior to analysis, films were coated with gold to make the samples conductive. Subsequently, samples were observed at 1000× magnification.

### 2.4. Film Thickness

Film thickness was measured using a hand-held digital micrometer (51031 Käfer, Villingen-Schwenningen, Germany). Measurements were carried out at different film locations and the mean thickness value was used to calculate the permeability of the films.

### 2.5. Colour Measurement

The surface colour of gelatin films was measured using a Minolta chromameter (CR-300, Minolta Camera Co., Osaka, Japan). Gelatin films were placed on the surface of a white standard plate (*L* = 97.79, *a* = 5.18, *b* = 7.91) and Hunter *L*, *a* and *b* colour values were measured. Colour coordinates ranged from *L* = 0 (black) to *L* = 100 (white), −*a* (greeness) to +*a* (redness), and −*b* (blueness) to +*b* (yellowness).

### 2.6. Film Opacity

The opacity of gelatin films was determined using a spectrophotometer (Cary 300 Bio, UV-Vis Spectrophotometer, Varian Instruments, CA, USA), set at a wavelength of 500 nm. Four film specimens were taken from each film sample and cut into rectangular pieces (45 × 10 mm). The sample was placed on the inner side of a transparent plastic 10 mm cuvette and the absorbance measured.

The opacities of films were calculated by the following equation according to the method described by Gontard *et al.* [26]:

opacity = absorbance at 500 nm × film thickness(1)

### 2.7. Mechanical Properties

The mechanical properties of films were evaluated and included; tensile strength (TS), elongation at break (EAB) and puncture strength (PS) using an Imperial 2500 Mecmesin force and torque tester (Mecmesin Ltd., Slinfold, West Sussex, England) according to the ASTM-D882 [27]. TS of a film is the maximum stress that a film can take before breaking, meanwhile EAB is the percentage increase in length of the film before the point of break and PS is the maximum stress required to rupture or penetrate the film. The films were cut into strips (100 × 25.4 mm) prior to analysis.

### 2.8. Water Vapour Permeability (WVP)

Water vapour permeability (WVP) was calculated from the following equation:

WVP = (quality of permeant/time) × (film thickness/film area × pressure difference)(2)

WVP of gelatin films was measured according to the WVP correction method of McHugh *et al.* [28] which is a modification of the ASTM E-96 standard method [29] for determining WVP of synthetic packaging materials. Perspex circular WVP cups were manufactured according to the specifications of McHugh *et al.* [28]. Distilled water (6 mL) was added into the each test cup and film samples were placed over the circular opening, tightened and secured in place using silicon grease. The cups were maintained under controlled conditions of humidity and temperature (50% ± 5% RH and 23 ± 2 °C). The weight loss from the samples with 5 replicates was monitored for 10 h period with weights recorded at 1 h intervals.

### 2.9. Oxygen Permeability (OP)

Oxygen permeability was conducted according to the method developed by Papkovsky [30] and Wang *et al.* [31]. An oxygen sensor was placed inside the test chamber and the composite film was then mounted between the upper lid and lower cup (the two halves of the test chamber) and fixed tightly using screws. Nitrogen gas was blown into the chamber through one pipe, while the other pipe was opened to evacuate the chamber until the nitrogen reading became stable. Both pipes were then shut. The oxygen sensor measured the increase in oxygen content over time during the testing period. The graphed data was evaluated using the developed equation:

OP = [*S*/(60 × β)] × (*V*/20.5) × (273/298) × [(*T* × 1000)/*A*]/101.625 × 10^9^/24 (3)

Where OP = oxygen permeability (cm^3^·μm/m^2^·day·kPa); *S* = slope indicating the transmission rate of oxygen; β = permeability coefficient (4.776), a constant value as all treatments were conducted at the same conditions; *A* = surface area of the film (m^2^); *T* = thickness of the test film samples (μm); *V* = volume of the chamber (mL).

### 2.10. Water Solubility of Gelatin Films

The film solubility was determined according to the method of Gontard and Guilbert [32] by trimming the samples into small strips. Small film strips were dried in an oven (Memmert ULM 500, Schwabach, Germany) at 100 °C for 24 h to a constant weight. Each dried sample was immersed in 100 mL of distilled water for 24 h. Film samples were then removed from solution and re-dried at 100 °C for 24 h. Final weights were recorded and solubility calculated as:

solubility = [(initial weight − final weight)/initial weight] × 100%(4)

### 2.11. Attenuated Total Reflectance-Fourier Transform Infrared (ATR-FTIR) Spectroscopy

The IR spectra for gelatin films were determined using a Varian 600-IR Series FTIR (Varian Resolutions, Varian Inc, Victoria, Australia) equipped with horizontal attenuated total reflectance (ATR) ZnSe cell at room temperature. The detector used was a Deuterated Tri-Glycine Sulfate (DTGS-KBR). Before film analysis, a background spectrum using a clean crystal cell was recorded. Films were placed onto the crystal cell and the cell was clamped into position on the FTIR spectrometer. FTIR spectra were recorded in the range of 500–4000 cm^−1^ with automatic signal gain collected in 32 scans with a resolution of 4 cm^−1^ that were rationed against a background spectrum. Four replicate spectra were obtained and the average spectrum was taken for analysis. 

### 2.12. Statistical Analysis

Statistical analyses were performed using one-way analysis of the variance (ANOVA) and the LSD test (least significant difference) which showed the statistically different values. Statgraphics Centurion XV software programme (statPoint Inc., Warrenton, VA, USA) was used with differences at *p* < 0.05 were considered to be significant. Differences between means were compared using Duncan’s multiple range test method.

## 3. Results and Discussion

### 3.1. Film Morphology

The surface micrographs obtained by SEM are shown in Figure 1. The results demonstrated that the microstructure of gelatin films with CO were compact but contained some bubbles and oil droplets. The images also showed that as the concentration of gelatin increased, the oil droplets were more intense on film surfaces resulting in a more noticeable irregular surface. The microstructure of films obtained suggested that there might be a decrease in the moisture barrier properties of films due to the presence of some bubbles and oil droplets. However, a dense film matrix was observed as gelatin content increased, indicating that an interaction was formed in the presence of CO, which became homogeneously entangled with gelatin molecules, with CO appearing to act as a filling substance in the gelatin network [6].

**Figure 1:** SEM images of composite films derived from beef, pork and fish gelatin sources with the concentrations of 4% (**a**–**c**), 6% (**d**–**f**) and 8% (**g**–**i**).

### 3.2. Film Thickness

The film thickness of all gelatin composite films increased (*p* < 0.05) when gelatin concentrations of 6% and 8% were utilized (Table 1). When comparing the results of this study with that of Nur Hanani *et al.* [25], gelatin films containing CO (composite films) had increased film thicknesses. The results obtained are in agreement with data generated in other studies [4,33,34] which suggested that edible films incorporated with hydrophobic substances, such as waxes and oils, form thicker films due to the higher water content present in lipid-emulsified films.

**Table 1:** Mechanical properties of gelatin films.

Samples	Thickness (μm)	Tensile Strength (MPa)	Puncture Strength (N)	Elongation (%)
*4%*				
Beef	63.73 ± 8.31 ^d^	4.23 ± 0.88 ^f^	10.00 ± 1.61 ^d^	101.38 ± 9.92 ^c, d^
Pork	63.80 ± 3.94 ^d^	6.05 ± 0.19 ^e^	11.79 ± 0.21 ^c, d^	109.60 ± 11.53 ^c^
Fish	65.77 ± 2.90 ^d^	4.84 ± 0.11 ^f^	11.51 ± 1.10 ^c, d^	184.81 ± 4.91 ^a^
*6%*				
Beef	85.13 ± 1.94 ^c^	2.41 ± 0.54 ^g^	12.69 ± 0.86 ^c^	141.04 ± 16.27 ^b^
Pork	55.10 ± 1.93 ^d^	7.59 ± 0.45 ^c^	20.68 ± 0.77 ^b^	93.37 ± 11.37 ^d^
Fish	66.87 ± 6.12 ^d^	6.56 ± 0.31 ^d, e^	20.15 ± 2.01 ^b^	139.78 ± 13.44 ^b^
*8%*				
Beef	115.71 ± 3.73 ^a^	7.01 ± 0.69 ^c, d^	20.43 ± 2.44 ^b^	192.34 ± 11.86 ^a^
Pork	104.47 ± 7.71 ^b^	8.96 ± 0.26 ^b^	22.88 ± 0.76 ^a^	115.18 ± 8.26 ^c^
Fish	109.70 ± 5.77 ^a, b^	11.14 ± 0.84 ^a^	22.14 ± 2.16 ^a, b^	114.28 ± 7.79 ^c^

Means in the same column followed by the same letter are not significantly different (*p* < 0.05).

### 3.3. Colour Attributes and Opacity of Gelatin-Based Composite Films

The colour attributes of gelatin composite films derived from beef, pork and fish sources are presented in Table 2. Results demonstrated that different gelatin sources used to manufacture composite films affected (*p* < 0.05) the *L* values, with films derived from pork gelatin sources possessing the highest *L* value. Results also indicated that increasing the concentration of gelatin decreased (*p* < 0.05) the *L* value of composite films manufactured from gelatin derived from beef sources. Composite films derived from beef gelatin sources also had lower (*p* < 0.05) *a* values compared to those derived from pork and fish gelatin sources.

**Table 2:** Colour properties and opacity of gelatin films.

Samples	*L*	*a*	*b*+	Opacity
*4%*				
Beef	93.23 ± 0.08 ^b^	−1.45 ± 0.04 ^e^	8.41 ± 0.13 ^b^	18.31 ± 0.37 ^i^
Pork	93.75 ± 0.04 ^a^	−1.09 ± 0.03 ^b, c^	5.94 ± 0.07 ^c, d^	22.19 ± 0.05 ^h^
Fish	90.80 ± 0.55 ^e^	−0.84 ± 0.07 ^a^	5.82 ± 0.07 ^c^	41.43 ± 0.03 ^d^
*6%*				
Beef	92.40 ± 0.17 ^c^	−1.65 ± 0.02 ^f^	9.67 ± 0.06 ^a^	40.27 ± 1.14 ^e^
Pork	93.80 ± 0.04 ^a^	−0.82 ± 0.03 ^a^	5.32 ± 0.03 ^e^	22.75 ± 0.13 ^g^
Fish	92.54 ± 0.30 ^c^	−0.89 ± 0.06 ^a^	5.52 ± 0.05 ^e^	50.80 ± 0.01 ^b^
*8%*				
Beef	91.80 ± 0.41 ^d^	−1.31 ± 0.14 ^d^	8.35 ± 0.63 ^b^	47.25 ± 0.04 ^c^
Pork	93.88 ± 0.02 ^a^	−1.16 ± 0.03 ^c^	6.17 ± 0.03 ^c^	24.83 ± 0.15 ^f^
Fish	92.43 ± 0.02 ^c^	−1.01 ± 0.05 ^b^	6.01 ± 0.08 ^c, d^	103.9 ± 0.07 ^a^

Means in the same column followed by the same letter are not significantly different (*p* < 0.05).

Additionally, composite films manufactured using pork- and fish-derived gelatins did not significantly show differences in *b* values. However, composite films derived from beef gelatin sources possessed higher (*p* < 0.05) *b* values. This was most probably due to the base colour of beef gelatin powder which possessed a yellowish hue compared to the other gelatin powder sources. The results obtained also indicated a decrease in *L* and *a* values for all composite films when compared with gelatin films manufactured without the use of CO [25], regardless of the gelatin source used. However, the *b* values for all gelatin composite films were higher compared to those gelatin films manufactured by Nur Hanani *et al.* [25] which did not employ the use of CO. The yellowish hue produced in the gelatin composite films was as a result of using CO which had a yellowish colour. It is possible that this effect, if perceived as commercially negative, might be addressed by decolourising the oil, using colourising ingredients in the films or using similar but colourless oil variants.

Visually, all gelatin composite films containing CO were opaque (Figure 2). The results from spectrophotometer indicated that the addition of gelatin and CO into film-forming solutions led to increased (*p* < 0.05) opaqueness for all gelatin-based composite films (Table 2). This means opacity was strongly related to lipid migration during film preparation, which could be visualized as a cloudy appearance of the films [8]. Therefore, addition of lipids causes the films to lose or reduce their transparency [3,5,35,36,37].

**Figure 2:** Films manufactured from gelatin derived from (**a**) beef, (**b**) pork and (**c**) fish sources with the concentrations of 4%, 6% and 8%.

### 3.4. Mechanical Properties

The mechanical properties of gelatin composite films are shown in Table 1. The TS of composite films were significantly (*p* < 0.05) affected by gelatin source, particularly at concentrations of 6% and 8%, for example, composite films manufactured from beef gelatin at 6% and 8% possessed the lowest TS values of all composite films manufactured. The increased concentration of gelatin also increased (*p* < 0.05) the TS values of composite films derived from pork and fish gelatin sources with fish gelatin employed at an 8% concentration showing the highest TS value (11.14 MPa). This trend was also observed for all composite films when the EAB test was conducted. Differences in EAB values for all composite films were significantly (*p* < 0.05) dependent on the concentration of gelatin used, especially for those derived from beef gelatin. With respect to PS, composite films manufactured from gelatin derived from beef sources had the lowest PS value, regardless of the gelatin concentration used. The results also showed that no significant differences in PS values were found between composite films manufactured from gelatin derived from pork and fish sources. Statistical analysis also showed that increasing the concentration of gelatin increased (*p* < 0.05) the PS values of all gelatin composite films. 

When the composite films produced in this study were compared with pure gelatin films [25], results showed that composite films possessed greater flexibility. The increased flexibility observed in composite films may have resulted from CO molecules filling in the physical spaces naturally occurring within the gelatin protein network.

### 3.5. Water Permeability

The WVP of gelatin-based composite films incorporating CO is shown in Figure 3. Irrespective of gelatin source, gelatin concentrations of 4% and 8% did not significantly affect WVP values of composite films. However, at a 6% gelatin concentration, composite films manufactured from gelatin derived from beef sources had higher (*p* < 0.05) WVP values than composite films derived from fish gelatin sources. The results also demonstrated that increasing gelatin concentration from 4% to 8% increased (*p* < 0.05) the WVP values of all gelatin-based composite films. According to Nur Hanani *et al.* [25] and Hoque *et al.* [37], some gelatins have hydrophilic characteristics that allow the material to bind with water molecules and thereby encourage water vapour absorption. When the water barrier properties of composite gelatin-based films produced in this study were compared with pure gelatin films [25], it was found that the gelatin-based composite films had higher WVP values. This result contradicts what should have occurred as proposed by the film formulation model by Wang *et al.* [6].

**Figure 3:** Water vapour permeability values of composite films derived from beef, pork and fish gelatin sources with the concentrations of 4%, 6% and 8%. Error bars represent standard deviations of data with letters indicate significant differences (*p* <0.05) between the WVP values.

According to Bertan *et al.* [3], adding lipids to protein films can increase the hydrophobicity of the film matrix depending on the type and concentration of lipid employed. Accordingly, it is likely that the quantity of oil employed, rather than the oil type used, was responsible for the reduced WVP properties associated with the gelatin-based composite films produced in this study as it has been shown that CO used in protein-based films has previously decreased WVP values [4,6]. The level of CO used in this study may have also been responsible for the development of varying sizes of air bubbles in the composite films and these too might serve to reduce WVP barrier properties, by creating a less torturous path for water molecules to travel through the film.

### 3.6. Oxygen Permeability

Oxygen permeability of gelatin composite films is presented in Figure 4. Oxygen permeability values for all gelatin-based composite films were not significantly different when gelatin was employed for film manufacture at a 4% concentration. At a 6% concentration, the oxygen permeability of composite films manufactured from gelatin derived from fish sources was significantly (*p* < 0.05) higher compared to films derived from beef and pork gelatin sources. Overall, increasing the concentration of gelatin in films increased (*p* < 0.05) OP. When the composite films manufactured in this study were compared with pure gelatin films [25] it was observed that composite films containing CO had decreased oxygen barrier properties for all films, with the exception of those produced using both pork and beef gelatin at a 6% concentration. 

**Figure 4:** Oxygen permeability values of composite films derived from beef, pork and fish gelatin sources with the concentrations of 4%, 6% and 8%. Error bars represent standard deviations of data with letters indicate significant differences (*p* <0.05) between the oxygen permeability values.

The increased OP observed in composite films may in fact be related to the significant presence of CO (highest concentration of oil use in such films to date) and the hydrophobic nature of this lipid component, consequently facilitating oxygen transfer [3,6,37,38]. Similar trends were also observed by Bertan *et al.* [3] when hydrophobic substances (up to 10% of gelatin) were added to the gelatin and triacetin films. These authors suggested that this behavior was caused by the formation of microscopic holes in the film structure. Interestingly, their suggestion is supported by evidence determined in this study on the presence of similar air bubbles in our own gelatin-based composite films (as previously shown in SEM images). Even with this increase in OP, all gelatin composite films produced in this study still had lower permeability values when compared with other studies [3,39], in spite of the amount of CO used, which was much greater (55.18% of gelatin powder used).

### 3.7. Water Solubility

The solubility of gelatin-based composite films is presented in Figure 5. The results demonstrated that as gelatin concentration increased from 4% to 8%, there were increases (*p* < 0.05) in film water solubility values for composite films derived from fish gelatin. However, these films had the lowest solubility values when compared to composite films derived from beef and pork gelatin sources, regardless of concentration used. At a gelatin concentration of 4%, no significant differences in the water solubility of composite films were determined between those formed from both beef and pork gelatin. When compared with the pure gelatin films [25], the addition of CO had caused an increase (*p* < 0.05) in the water solubility of the films particularly for composite films derived from pork and fish gelatin sources. According to the scientific literature, Gontard *et al.* [40] and Bertan *et al.* [3] obtained similar results with composite gelatin and gluten plus lipid films. Meanwhile, Pérez-Mateos *et al.* [1] observed that the higher the oil concentration in the film, the lower the protein fraction present in the soluble matter, probably because of an complexing interaction between the protein and the oil in the film resulting in protein insolubilization.

**Figure 5:** Water solubility values of composite films derived from beef, pork and fish gelatin sources with the concentrations of 4%, 6% and 8%. Error bars represent standard deviations of data with letters indicate significant differences (*p* <0.05) between the water solubility values.

However, contrary results were obtained for composite films manufactured from gelatin derived from beef sources. At a 6% gelatin concentration, films derived from beef gelatin sources had the highest water solubility. This was most likely due to the presence of lactic acid usage which was added during the preparation of the solution to control the pH at 10.54. During the preparation of film forming solutions, lactic acid had been used in the solutions of beef gelatin sources at 6% concentration to adjust the pH value. Lactic acid is hygroscopic, therefore it had attracted and held water molecules and encourage solubility of film in water.

### 3.8. FTIR Spectroscopy

FTIR analysis was carried out on all composite films (Figure 6). The absorption bands for gelatin-based composite films containing CO in the IR spectra are situated in the amide band region. The band situated around 3299, 1635, 1550, 1238 cm^−1^ correspond to amide-A and water molecules, amide I, amide II, and amide III, respectively [41,42,43]. Amide-A represents NH-stretching coupled with hydrogen bonding; amide-I represents C = O stretching/hydrogen bonding coupled with COO; amide-II arises from the bending vibration of N–H groups and stretching vibrations of C–N groups; amide-III is related to vibrations in the plane of C–N and N–H groups of bound amide or vibrations of CH_2_ groups of glycine [40,42,43].

**Figure 6:** FTIR spectra of composite films derived from (**a**) beef, (**b**) pork and (**c**) fish sources with different concentration in the range of 4000–500 cm^−1^.

Among these absorption bands, the amide I band between 1600 and 1700 cm^−1^ is the most useful peak for infrared analysis of secondary protein structures like gelatin [44,45]. Jongjareonrak *et al.* [40] and Yakimes *et al.* [46] reported that the absorption peak at 1633 cm^−1^ is characteristic for the coil structure of gelatin. Increasing gelatin concentrations, particularly for films manufactured from gelatin derived from pork and fish sources, shifted the amide I peak to a higher wavenumber. The change in amide I band for gelatin films suggested that CO might affect the helix coil structure of gelatin films as suggested by Jongjarenrak *et al.* [40]. These authors also found that the wavenumber for amide I shifted due to the presence of substances like BHT and α-tocopherol in films derived from fish gelatin sources. Additionally, the Amide A band for gelatin composite films derived from pork and fish sources also shifted to a higher wavenumber. 

The FTIR spectra of the films also showed some interactions occurred between gelatin and CO as indicated by the presence of a high peak in the frequency range between 2500 and 3100 cm^−1^. The peaks around 2925 and 2854 cm^–1^ are related with the symmetric and asymmetric stretching vibration of the aliphatic group (CH_2_) [7,47]. Meanwhile, a peak around 1745 cm^−1^ also appeared and indicated strong C = O absorption from the oil. Composite films manufactured from gelatin derived from beef sources with 6% concentration displayed a higher wavenumber of 1116 cm^−1^ compared with other gelatin films. The peak shift is most likely due to the presence of lactic acid which was used during the preparation of the solution to standardize pH solution values. This spectrum supports previously described results, for example, the increased solubility of composite beef gelatin derived films due to the presence of lactic acid.

## 4. Conclusions

Experimental studies were conducted and based on the proposed model for optimum gelatin-based composite film manufacture as outlined by Wang *et al.* [6]. This model proposed that the optimum level of lipid (CO) that should be added to film forming solutions was 55.18%. This amount of lipid is higher than that used in previous and related studies. The addition of this lipid led to increased opaqueness for all gelatins composite films and also resulted in increased film flexibility. However, adding the higher amount of lipid to pure gelatin films did not assist in improving the water barrier properties of the gelatin-based composite films. In terms of oxygen permeability, oil addition also decreased gas barrier properties (when compared with pure gelatin films), however, it is noteworthy that all gelatin-based composite films produced as part of this research, had lower oxygen permeability values when compared with other studies. FTIR analysis revealed that specific interactions occurred between gelatin and CO. From this study, it is clear that further improvements are required to enhance the general barrier properties of gelatin-based composite films and further investigation needs to focus on increasing the interaction between protein and lipid components within and throughout the film structure.
